# Hybrid Diagnosis Models for Autism Patients Based on Medical and Sociodemographic Features Using Machine Learning and Multicriteria Decision-Making (MCDM) Techniques: An Evaluation and Benchmarking Framework

**DOI:** 10.1155/2022/9410222

**Published:** 2022-11-16

**Authors:** M. E. Alqaysi, A. S. Albahri, Rula A. Hamid

**Affiliations:** ^1^Informatics Institute for Postgraduate Studies (IIPS), Iraqi Commission for Computers and Informatics (ICCI), Baghdad, Iraq; ^2^Department of Medical Instruments Engineering Techniques, Al-Farahidi University, Baghdad 10021, Iraq; ^3^College of Business Informatics, University of Information Technology and Communications (UOITC), Baghdad, Iraq

## Abstract

**Method:**

The three-phase framework integrated the MCDM and ML to develop the diagnosis models and evaluate and benchmark the best. Firstly, the new ASD-dataset-combined medical tests and sociodemographic characteristic features is identified and preprocessed. Secondly, developing the hybrid diagnosis models using the intersection process between three FS techniques and five ML algorithms introduces 15 models. The selected medical tests and sociodemographic features from each FS technique are weighted before feeding the five ML algorithms using the fuzzy-weighted zero-inconsistency (FWZIC) method based on four psychiatry experts. Thirdly, (i) formulate a dynamic decision matrix for all developed models based on seven evaluation metrics, including classification accuracy, precision, F1 score, recall, test time, train time, and AUC. (ii) The fuzzy decision by opinion score method (FDOSM) is used to evaluate and benchmark the 15 models concerning the seven evaluation metrics.

**Results:**

Results reveal that (i) the three FS techniques have obtained a size different from the others in the number of the selected features; the sets were 39, 38, and 41 out of 48 features. Each set has its weights constructed by FWIZC. Considered sociodemographic features have been mostly selected more than medical tests within FS techniques. (ii) The first three best hybrid models were “ReF-decision tree,” “IG-decision tree,” and “Chi^2^-decision tree,” with score values 0.15714, 0.17539, and 0.29444. The best diagnosis model (ReF-decision tree) has obtained 0.4190, 0.0030, 0.9946, 0.9902, 0.9902, 0.9902, 0.9902, and 0.9951 for the C1=train time, C2=test time, C3=AUC, C4=CA, C5=F1 score, C6=precision, and C7=recall, respectively. The developed framework would be beneficial in advancing, accelerating, and selecting diagnosis tools in therapy with ASD. The selected model can identify severity as light, medium, or intense based on medical tests and sociodemographic weighted features.

## 1. Introduction

Autism spectrum disorder (ASD) is a neurodevelopmental disorder that impairs an individual's social, communication, and learning abilities [1], in addition to restriction, repetitive patterns of behavior, interests, or activities. This disease begins in childhood and may last for life. Many children suffer from this disease, which greatly affects their behavior [2]. ASD affects families in terms of the pressure parents are exposed to their son, whether psychological or material (money). In contrast, the cost of treatment for this disease is expensive. Leo Kanner described autism disease for the first time in 1943, attempting to comprehend the association between autism and sociodemographic characteristics, including socioeconomic class, sex, maternal education, age, and race [3]. Every year, the World Health Organization (WHO) diagnoses autism globally in one out of every 160 children [4, 5].

The introduction of the presented study has discussed five important questions and provided the appropriate answers.

The first question is, “What are ASD diagnoses and symptoms?”

Psychiatric diseases are considered one of the most difficult types in the diagnosis process due to the overlap in symptoms resulting from the lack of experience and experts in this field. Nonetheless, doctors and medical personnel regard the diagnosis of autism in children in their first two years to be a difficult undertaking. Although there are several clinical tests for the early detection of ASD, they are complex diagnostics that are rarely utilized unless there is a considerable risk of developing ASD [6]. In contrast, the diagnosis of autism can occur at any age of the patient. Early detection helps to recover faster and significantly reduces the consumption of resources such as time and money [7]. One of the challenges researchers face is consuming time and money in diagnosing autism. The symptoms of autism differ from one patient to another. In addition, the disease's severity is different [8]. Clinical symptoms are different, such as fluttering, isolation of the patient from others, and lack of speech and interaction.

On the other hand, these symptoms can be observed through the Autism Diagnostic Observation Schedule (ADOS) and Autism Diagnostic Interview-Revised (ADI-R) questionnaires related to the behavior and action of the child [9, 10]. As mentioned above, there is an essential need for a method or tool that contributes to the autistic diagnosis process. So, the second question should be discussed: “How can ML and AI techniques benefit the ASD diagnosis process?”

ML and AI techniques play an important role in the diagnosis process contributing to early ASD diagnosis and providing excellent support for controlling and treatment [11–13]. In addition, after considerable advancements in computer science and information technology, ML is being used to detect and assess a variety of illnesses, such as lung cancer, hepatitis, heart disease, COVID-19, and diabetes [14–19]. ML models classify and predict various medical fields effectively. Several methods of ML have also been used for the diagnosis of ASD, such as random forest (RF), naive Bayes, and *K*-nearest neighbor (KNN), and deep learning, such as methods of recurrent neural network (RNN) and convolutional neural network (CNN). However, researchers face a lack of accuracy in diagnosing autism and nonoptimal data selection in ASD diagnosis regarding the affected features. Therefore, ML and AI techniques should continue to make more contributions to diagnosing autism based on the new datasets adopted in this research path. The third question must be presented: “What are the research directions for ASD diagnosis in the literature review based on AI and ML?”

Various trends have arisen in recognizing, diagnosing, and evaluating autism using AI and ML. First, magnetic resonance imaging (MRI) is a cross-sectional scan of the brain and a medical imaging technique that reveals pathological alterations in live tissues [20]. MRI is involved in diagnosing many wide diseases. Despite its effectiveness in the diagnosis process, it needs financial resources because of the high price of devices and manufacturing. In addition, not all hospitals have MRI devices, especially in remote and rural areas. Second, the electroencephalogram (EEG) employs small metal discs (electrodes) implanted in the scalp; this test monitors the electrical activity in the brain. Poor spatial resolution is the primary drawback of EEG recordings [21, 22]. In addition, it does not provide the maximum diagnostic accuracy for ASD. Besides, this path requires a specialist doctor with a long experience to give a correct result in the diagnosis process. Third, sociodemographic diagnosis is based on sociodemographic features (i.e., sex, age, and race) and can depend on ADOS and ADI-R that notes the behavior of the patient [5, 9, 10].

In conclusion, each diagnostic approach has limits concerning the employed diagnostic characteristics. Each technique alone does not give a reliable diagnosis procedure. These instructions could not have been carried out if the right diagnostic procedure had focused on certain characteristics while ignoring others. Accordingly, medical tests have a role in the diagnosis of utmost diseases. The integration of medical tests and sociodemographic features should be considered in the diagnosis process. Despite the above, little attention has been given to medical tests among sociodemographic features for ASD diagnosis in any research direction. Here, the fourth important question must be discussed: “What is the current scenario of literature for the diagnosis of ASD using sociodemographic and medical test features?” It needs to be further answered.

In the study of [6], authors utilized early detection ASD datasets of different stages of life (toddler, child, adolescent, and adult) and had used different feature selection (FS) such as correlation feature selection, gain ratio, information gain (IG), and ReliefF (ReF). In addition, they utilized different ML like decision tree, support vector machine (SVM), and AdaBoost. The features of a dataset are based on sociodemographics and use of feature transformation (Logarithmic, ZScore, Sine) then evaluation by various metrics such as classification accuracy (CA), sensitivity, specificity, area under curve (AUC), Kappa statistics, and Logloss. In the study by [23], detection of ASD was attempted using ML and deep learning techniques such as logistic regression (LR), SVM, naive Bayes, KNN, ANN, and CNN. Also, the features of the dataset are based on sociodemographics only. The applied metrics are CA, specificity, and sensitivity to evaluate the developed model. In the study [24], the adultization of different ML included AdaBoost, KNN, and ID3 with FS techniques such as correlation feature selection, gain index, IG, fast correlated-based filter, and Chi-Squared (Chi^2^). They were then evaluated by metrics: CA, specificity, sensitivity, and AUC. The authors in [25] deal with the data imbalance technique applied to the demographic ASD dataset using naive Bayes, decision tree (c4.5), RIPPER, and RF. Also, the study used methods such as the synthetic minority oversampling technique (SMOTE), random oversampling (ROS), and random undersampling (RUS) to achieve data balance and were evaluated by metrics such as specificity, sensitivity, Matthews' correlation coefficient, F1 score, false positive rate, precision, and AUC. In [26], diagnosis of ASD based on resampling techniques methods of resampling techniques to a normal distribution of ASD data improved accuracy in the prediction of autism and avoids the problem of data heterogeneity. The authors used naive Bayes, and RF with SMOTE, ROS, and RUS to achieve data balance then evaluated by CA, specificity, sensitivity, and receiver operating characteristics (ROC). In the study of [27], children between the ages of 4 and 11 were diagnosed with ASD using the categorization approach with 19 sociodemographic features. For classification, the linear discriminant analysis (LDA) and KNN algorithms are employed then evaluated by metrics such as CA, F1 score, and precision. The authors of [28], dealt with the diagnosis and prediction of autism using decision tree algorithm based on medical and family characteristics, therefore facilitating access to ASD knowledge and supporting professionals and physicians in their clinical decisions by An Ontology-Driven Decision Support for Autism Diagnosis and Treatment, and were evaluated by various metrics such as CA, specificity, and sensitivity. The data attributes are categorized under 13 categories: (1) diagnostic history, (2) review of systems, (3) prenatal/early postnatal history, (4) pulmonary, (5) developmental history, (6) hematologic, (7) endocrine/metabolic, (8) cardiovascular, (9) gastrointestinal, (10) current medications, (11) mental health, (12) genetic, and (13) immunologic.

The above literature shows a variance in feature selection techniques, machine learning algorithms, and performance evaluation metrics. In addition, selecting the developed optimal model for accurate ASD diagnosis is challenging. However, no study has been presented for evaluating and benchmarking the developed hybrid diagnosis models for selecting the best one, which is the study's aim. There are three main issues facing this aim. The first issue concerns the importance of ASD features, especially since most literature studies have not elaborated on important features that affect model classification. In light of whether the features are highly relevant or less, the second issue, evaluation metrics, is faced. In other words, the studies demonstrate diversity in evaluating the model performance by using some metrics as criteria and ignoring others. Their assessment is varied for designing and implementing an accurate diagnosis models. Accordingly, the evaluation metrics of the classification models are still comparative. They overlap with other models for multievaluation criteria, trade-offs, and criteria importance categorized under complex multicriteria decision-making (MCDM) problems. For the third issue about dataset availability, perhaps the most important challenge faced by most researchers is the lack of special integrated sociodemographic and medical test features in providing an efficient model for diagnosing autism. Besides, the number of ASD features used for diagnosing autism in the literature varies, and there is no precise justification for using some features and neglecting others. Therefore, the presented study used an integrated ASD dataset with sociodemographic and medical test features.

The last question to be discussed is, “What is the useful solution to select the best diagnosis model of ASD by integrating medical tests and sociodemographic features?”

The FS process benefits appear in selecting the ML model, which gives high diagnostic accuracy. The development of the diagnosis ML model concerning the selection of ASD features plays an important role in choosing the optimal special diagnosis model based on the approach used or the techniques. In the process of identifying features' importance, each of the features has a different significance. Accordingly, the filter approach performs the FS step as preprocessing before the learning step without involving a learning algorithm. The filter is independent of the learning algorithm and relies on underlying attributes of data [29]. In addition, popular ML algorithms can enhance the diagnosis of ASD and can match the new hybrid diagnosis model using exhaustive and best-researched algorithms. These algorithms include decision tree [30], naive Bayes [31], KNN [32], SVM [33], and AdaBoost [34]. The algorithms used are very realizable due to their great precision and adaptability for obtaining superior outcomes.

On the other hand, MCDM is defined as “an extension of decision theory that encompasses all decisions with numerous objectives. A technique for evaluating options based on distinct, sometimes contradictory criteria and merging them into a single overall evaluation” [35, 36]. MCDM is an umbrella term for a collection of formal techniques that strive to explicitly account for many factors when assisting individuals or groups in evaluating important decisions [37–39]. Numerous subjective weighting methods have been proposed; however, when it comes to weighting criteria, the analytic hierarchy process (AHP) [40–44] and best-worst method (BWM) [45, 46] methods have a high success rate. Nonetheless, the inconsistency issue of their weighing techniques has been addressed [17, 37, 47–51]. Therefore, the fuzzy-weighted with zero-inconsistency (FWZIC) method has been introduced [52]. FWZIC can assign weights for each set of medical tests and sociodemographic features resulting in each FS with zero inconsistencies regardless of the number of features. FWZIC computes and calculates the weight coefficient values of each feature separately and accurately to attain zero consistency. Compared to zero pairwise comparisons, FWZIC eliminates the potential for mistakes. Recently, the FWZIC method acquired attention and has been used in several studies [13, 53–56]. FWZIC method can process zero inconsistency. In addition, other MCDM methods can process the ranking issues using the fuzzy decision by opinion score method (FDOSM). This method is utilized for selecting the best rank (best solution). FDOSM utilized an ideal/optimal solution concept, eliminated inconsistency and two preferences, decreased the number of comparisons, provided fair and implicit comparisons, and needed fewer mathematical operations. In addition, it addressed the normalization and weight concerns that plagued MCDM techniques. FDOSM attempts to deal with ambiguous and fuzzy data by employing triangular fuzzy numbers (TFNs). The FDOSM technique offered a mathematical model to address MCDM issues involving a single context of decision-making followed by a group context of decision-making and has been used in [49, 54, 57].

This research paper presents a clear conception of the diagnosis of autism. This study led to a solution to the research gap for ASD diagnosis to present a dataset of medical tests integrated with sociodemographic features. In this study, the combination of medical tests and the sociodemographic behavior of the patient give a strong solution to increase the diagnosis procedure. The main objective is to develop a new framework for selecting the optimal diagnostic model capable of identifying autism severity levels such as light, medium, or intense. In this regard, the study contributions can be summarized in the following points:

(1) Develop hybrid diagnosis models for ASD patients based on medical tests and sociodemographic characteristic features by
  - Intersection process between three FS techniques and five ML algorithms
  - Construct weights for each set of FS techniques based on specialized psychiatry experts using the FWIZC method
  - Develop 15 hybrid diagnosis models based on the weighted dataset
(2) Develop an MCDM framework to evaluate and benchmark the 15 hybrid diagnosis models using the FDOSM method

## 2. Research Methodology

The research methodology can discuss the direction of the study in three phases. Firstly, the data identification and preprocessing, after that, the second phase is the development of hybrid diagnosis Models. Finally, the third phase is the evaluation and benchmarking framework.  Figure 1 illustrates the methodology of the study.

### 2.1. Phase 1: Data Identification and Preprocessing

The data obtained is real data from a diploma study at the Informatics Institute for Postgraduate Studies (IIPS). These data consist of 49 sociodemographic and medical test features and 538 patients. Besides, the “severity” feature is considered the class that includes three categories of labels: light, medium, and intense. The features are described in Table 1.

#### 2.1.1. Data Coding and Cleaning

For any data, removing any unknown symbols or outliers should be addressed. Therefore, converting text or string data to numeric data must be achieved due to the ML method dealing with numeric data. In the ASD dataset, data cleaning eliminates all unnecessary symbols such as “?”, “/”, and “-”.

#### 2.1.2. Imputing Missing Values

The used ASD dataset contains some missing values.  Figure 2 shows the percentage of missing values. Several methods can be used for filling in missing values and manipulating them, such as model-based imputer (simple tree), distinct value, a random value, or mean, which is the most frequently used for handling this type of data using Equation (1). Then, the dataset should be normalized because the data have different scales, as presented in the next section.

(1) $$\begin{array}{c} \text{Mean}=\frac{\text{sum}\left(\text{zi}\right)}{\text{count}\left(\text{zi}\right)}. \end{array}$$

#### 2.1.3. Dataset Normalization

Normalization is an operation that either modifies or rescales raw data such that each characteristic contributes uniformly. It addresses two primary data concerns that impede the learning process of ML algorithms: the existence of dominating features and outliers since the dataset has a different scale that can affect the model's process. This study used the min–max normalization approach to the ASD dataset, as seen in Equation (2).

(2) $$\begin{array}{c} x^{\prime }=\frac{x-\min\left(x\right)}{\max\left(x\right)-\min\left(x\right)}. \end{array}$$

#### 2.1.4. Data Imbalance

One important thing that some researchers overlook is data asymmetry. Consequently, models are biased, and accuracy can no longer be used to measure integrity. There are three classes of health conditions in the used dataset, as shown in Figure 3. Class (1) has 259 instances as “medium,” class (0) has 241 instances as “light,” and class (2) has 38 instances as “intense.”

An imbalance can be noticed in the used dataset, which can minimize the diagnosis process's accuracy. The SMOTE method commands resampling techniques utilized in ML to balance data based on the target class. In this context, the developed ML models can achieve high accuracy in classification and give a perception closer to reality [58]. SMOTE, a frequent oversampling technique, produces “synthetic” observations in the sample rather than duplicating data. This technique leverages the *K*-nearest neighbors of an observation to generate random synthetic observations [25]. At this step, the preprocessing stages have been stated and prepared for the ASD dataset to develop the hybrid models as presented in the next phase.

### 2.2. Phase 2: Development of Hybrid Diagnosis Models

This section addresses the stages of developing the hybrid diagnostic models for ASD.

#### 2.2.1. FS Approaches

FS approaches ease significant concerns in classification procedures as they enhance classification accuracy, reduce data dimensionality, and remove unnecessary data.  Figure 4 shows three filter approach methods: Chi^2^, IG, and ReF.

Each method of feature selection obtains a size different from the others. Furthermore, FS is considered essential in ML but does not always produce precision results due to not depending on expert judgment opinion. This stage chooses pertinent sociodemographic and medical tests, considers the class-labeled dataset, and scores these features based on their association with the class. Expert opinion plays an important role in the process of determining the importance of each feature. So that the importance of the influencer gives the subject a link from the feature that is irrelevant or has little influence on it to the feature that has very important; therefore, a modern MCDM method should be used for weights based on experts to overcome the above purpose. FWIZC method can handle this purpose, as presented in the next section.

#### 2.2.2. FWZIC

FWZIC is one MCDM method that needs to be used for weighting the features resulting from FS techniques (Chi^2^, IG, and ReF).  Figure 5 illustrates the steps of FWZIC through five essential processes that need to be applied for each set of medical tests and sociodemographic features resulting from three FS techniques [59]. The five steps are illustrated below.

**Step 1 .**

Establish the set of evaluation features: the predetermined set of assessment features of ASD is examined and presented in the first step.

**Step 2 .**

Structured expert judgment (SEJ): the identification and selection of expert team members from relevant fields of medicine (psychiatrists) are performed. Then, selection and nomination will commence. The SEJ panel has been formed.  Table 2 depicts the conversion of the linguistic scale to the corresponding numerical scale, which followed the development of an evaluation form to capture the consensus of all SEJ team members for each medical test and sociodemographic feature. A panel of four experts assesses the features subjectively, as illustrated in the following step.

**Step 3 .**

Building the expert decision matrix (EDM): the preceding stage defines the list of selected experts and each expert's choice within a specific feature. This stage builds the EDM. As stated in Table 3, the primary components of the EDM are the alternatives and decision criteria. Each criterion (Cj) in the attribute (represents the patient's features) crossovers with each selective expert (Ei) (represents the psychiatrist (who has evaluated the appropriate degree of relevance for each feature.

**Step 4 .**

Application of a fuzzy membership function: the fuzzy membership function and accompanying defuzzification procedure are used for the EDM's data to improve the data's accuracy and usability for future analysis. However, in MCDM, the problem is ambiguous and imprecise since giving a specific preference rate to each criterion is impossible. “The benefit of employing the fuzzy technique is the use of fuzzy numbers rather than exact numbers to calculate the relative value of the feature (criteria) to handle situations that are imprecise and ambiguous” [60–62]. In fuzzy MCDM, triangular fuzzy numbers (TFNs) are the most prevalent sort of fuzzy numbers. *A* = (*a*.*b*.*c*) is used to signify TFNs. Due to their conceptual and computational simplicity, they are often utilized in real applications [63], as seen by the triangle membership in Figure 6.

The membership function (*x*) of TFN *A* is given by

(3) $$\begin{array}{c} \mu \;A\left(x\right)=\left\{\begin{array}{cc} 0, & \text{if }x<a,\\ \frac{x-a}{b-a}, & \text{if }a\leq x\leq b,\\ \frac{c-x}{c-b}, & \text{if }b\leq x\leq c,\\ 0, & \text{if }x>c, \end{array}\right.\;\text{where }a\leq b\leq c. \end{array}$$

**Remark 1 .**

Let $\tilde{x}=\left(a1,b1,c1\right)$ and$\;\tilde{y}=\left(a2,b2,c2\right)$ be two nonnegative TFNs and ∈ℝ_+_. Following the extension principle, the arithmetic operations are defined as follows:

(4) $$\begin{array}{c} \tilde{x}+\tilde{y}=\left(a1+a2,b1+b2,c1+c2\right),\\ \tilde{x}-\tilde{y}=\left(a1-c2,b1-b2,c1-a2\right),\\ \alpha \tilde{x}=\left(\alpha a1,\alpha b1,\alpha c1\right),\\ \tilde{x}-1≅\left(\frac{1}{\text{c}1},\frac{1}{\text{b}1},\frac{1}{\text{a}1}\right),\\ \;\tilde{x}\times \tilde{y}≅\left(a1a2,b1b2,c1c2\right),\\ \frac{\tilde{x}}{\tilde{y}}≅\left(\frac{a1}{c2},\frac{b1}{b2},\frac{c1}{a2}\right). \end{array}$$

The value of each Numerical term with TFN is shown in Table 4.

Table 4 indicates that all linguistic variables be transformed to TFNs, supposing that the fuzzy number is the variable for each expert *N* feature (criteria). In other words, in psychiatry, expert *N* was tasked with identifying the critical degree of the assessment features (medical tests and sociodemographic) inside variables assessed using language variables.

1. By using Equation (5), the ratio of fuzzification data is determined. As demonstrated in Table 5, the preceding equations are employed with TFNs [63].

(5) $$\begin{array}{c} \frac{\tilde{\text{Imp}\left(E1/C1\right)}}{\sum_{j=1}^{n}\text{I}\text{mp}\left(E1/C_{1j}\right)}, \end{array}$$

where $\tilde{\text{Imp}\left(E1/C1\right)}$ represent the fuzzy number of Imp (*E*1/*C*1).

(2) To determine the final fuzzy values of the weight coefficients of the evaluation feature (criterion) ${\left(\tilde{w1},\tilde{w2},\cdots ,\tilde{\text{wn}}\right)}^{T}$, the mean values are determined. The fuzzy EDM $\left(\tilde{\text{EDM}}\right)$ is utilized to calculate the final weight value of each feature (criterion) using Equation (6).

(6) $$\begin{array}{c} {\tilde{w}}_{j}=\left.\left(\overset{m}{\underset{i=1}{\sum }}\frac{Imp\left(\tilde{E_{lj}}/C_{lj}\right)}{\sum_{j=1}^{n}Imp\left(\tilde{E_{lj}}/C_{lj}\right)}\right)/m\right),\text{for }i=1,2,3,..m\text{ and }j=1,2,3,..n. \end{array}$$

(3) *Defuzzification to find the final weight*: the centroid approach is the most prevalent defuzzification technique. Using TFNs, the mathematical expression for this procedure is (*a* + *b* + *c*)/3. Before computing the final values of the weight coefficients, the weight of importance should be allocated to each feature (criterion) based on the total weights of all features (criteria) for the rescaling purpose used in this step

**Step 5 .**

Computation of the final values of the weight coefficients of the evaluation criteria: in this stage, the final values of the weight coefficients for the evaluation feature (criteria) (*w*1, *w*2, ⋯,*w*48)^*T*^ that represented (C1=sex, C2=the blood type of the patient…. C48=mother age) are determined using the fuzzy data for the criterion from the previous step.

All five steps must be applied for each result of the FS technique. Besides, the sum of the weight must be equal to one. At this point and after calculating the weights for selected features (criteria), the constructed weights are distributed among the balanced ASD dataset for each FS technique value. Therefore, each weight generated must be multiplied by its fit data by using the following:

(7) $$\begin{array}{c} \text{ASD}=\overset{m}{\underset{i=1}{\sum }}B_{i}\left(W_{i}X_{i}\right)+\varepsilon , \end{array}$$

where *B*_*i*_: estimation parameter for feature *i*, *W*_*i*_: weight of feature *i*, and *ε*: error of estimation. After completing the process of Equation (7), the result is to produce a new weighted dataset for each FS technique that needs to be applied to the ML model in the next section.

#### 2.2.3. Construction of Hybrid ML Models

This section builds hybrid diagnosis models based on the intersection of five supervised ML algorithms and three FS techniques, as shown in Figure 7. The hybrid diagnostic models must be used for training and testing by combining ML algorithms with the FS techniques established in the previous section (weighted datasets). The five ML algorithms in our trials as possibly viable methods to enhance the diagnosis of ASD and to match the new hybrid diagnosis model using exhaustive and best-researched algorithms. The utilized ML algorithms are as follows: (1) decision tree, (2) naive Bayes, (3) KNN, (4) SVM, and (5) AdaBoost. The results of the intersection process introduced 15 hybrid diagnosis models. All the hybrid models need to be evaluated for their performance metrics, as explained in the next stage.

#### 2.2.4. Evaluation Criteria for the Hybrid Models

Measuring performance is essential for determining how effectively hybrid diagnosis models fulfill the objective. The performance of the 15 hybrid diagnosis models must be examined using five performance-evaluation metrics on the tested ASD datasets. Including CA, precision, F1 score, recall, and AUC. The metric criteria are defined and presented as follows:

1. *CA*: this is the commonly used metric for evaluating classification models; it quantifies the degree of closeness to the real value. Accuracy is computed by

(8) $$\begin{array}{c} \text{CA}=\frac{\text{TP}+\text{TN}}{\text{TP}+\text{FP}+\text{FN}+\text{TN}}. \end{array}$$

(2) *Sensitivity (TPR/recall)*: the number of successfully identified labels from all the positive representations. It might be viewed as the capacity of a test to distinguish people with a condition properly. Sensitivity is computed using this method:

(9) $$\begin{array}{c} \text{Recall}=\frac{\text{TP}}{\text{TP}+\text{FN}}. \end{array}$$

(3) *Precision*: it is the proportion of properly identified samples among all detected samples. It evaluates the classifier's capacity to exclude irrelevant topics. Precision is computed by

(10) $$\begin{array}{c} \text{Precision}=\frac{\text{TP}}{\text{TP}+\text{FP}}. \end{array}$$

(4) *F1 score*: it is the weighted average of recall and precision. The best F1 score value is 1, while the poorest one is 0. The contribution of precision and recall to the F1 score is equivalent. The F1 score is computed with the following:

(11) $$\begin{array}{c} \text{F}\_\text{score}=\frac{2*\text{TP}}{2*\text{TP}+\text{FP}+\text{FN}}. \end{array}$$

(5) *AUC*: the associated ROC curve is used to evaluate the classification model's performance at different threshold settings. The AUC displays the model's performance by differentiating between classes (i.e., a degree of separability). A greater AUC is preferable. With a higher AUC, the model can identify ASD samples with light, moderate, and intense severity
(6) *Training time*: it means the time the model takes to train the detection of ASD. The lower, the better, and vice versa
(7) *Time testing*: it means the time of model takes to test the process: the lower, the better, and vice versa

The developed models must be benchmarked to select the best one based on the five performance-evaluation metrics (criteria). Therefore, a new decision matrix needs to be developed for this purpose. In addition, another MCDM method (FDSOM) needs to be used to evaluate and benchmark all developed diagnosis models using the developed decision matrix, as explained in the next section.

### 2.3. Phase 3: Evaluation and Benchmarking Framework

This stage covers the development framework for evaluating and benchmarking the 15 hybrid ASD diagnostic models based on MCDM approaches. The first part covers the developed decision matrix (DM), while the second part explains the FDOSM method steps.

#### 2.3.1. DM

This section explains the developed dynamic DM used to evaluate and benchmark hybrid diagnosis models. DM is the most important aspect of the assessment and benchmarking technique [48, 54, 64–67]. The primary components of decision-making are choice criteria and alternatives. The evaluation criteria represent the metrics used to benchmark the 15 hybrid diagnostic models (representing the alternatives). The processes taken to construct the DM are detailed in Table 6.

#### 2.3.2. FDOSM Method for Ranking Hybrid ML Models

FDOSM is considered an MCDM method for ranking and evaluation benchmarking. In decision-making, FDOSM comprised three block units: the data input unit, the data transformation unit, and the data processing unit [68]. The framework for group decision-making consists of two phases: external and internal aggregations.  Figure 8 depicts the FDOSM methodology. The FDOSM steps can be expressed as follows:

- *Data input unit*: like existing MCDM approaches, the proposed MCDM method assigns *m* choices to each MCDM issue. *A*1, ⋯, Am that presented hybrid models and *n* set of decision criteria *C*1, ⋯, Cn that represented evaluation criteria. The DM represents this block's output. Next step, this choice matrix is converted into an opinion matrix [68].
- *Data transformation unit*: upon constructing the DM (the output of the first block), FDOSM adopts the transformation unit by selecting a three-parameter optimal solution (minimum, maximum, and critical values). The cost criterion combines the minimum value criterion, wherein the lowest value indicates the best option. The maximum value is used with the benefit criteria, whereby the highest value means the best solution. Critical value philosophy is the value employed in many situations, especially when the optimal answer is neither minimum nor maximum, as in the case of blood pressure. The following steps are outlined and detailed for this stage:

**Stage 1 .**

Choose the optimal solution. Consequently, the optimal solution is described as follows:

(12) $$\begin{array}{c} A*=\left\{\left[\left(\underset{i}{\max}v_{ij}\left|j\in J\right.\right),\left(\underset{i}{\min}v_{ij}\left|j\in J\right.\right),\left(Op_{ij}\in I.J\right)\left|i=1.2.3..\cdots \text{m}\right.\right]\right\}. \end{array}$$

**Stage 2 .**

Compare the optimum solution to alternative values based on the criterion. This method of allocating weights to assessment criteria is implicitly supplied. Subjectively, the significance of the differences between the ideal solution and the alternatives is evaluated as shown in

(13) $$\begin{array}{c} \text{O}{\text{p}}_{\text{Lang}}=\left\{\left(\left(\begin{array}{c} \tilde{v}\\ ij \end{array}⊗v_{ij}\left|j\in J\right.\right)\left|i=1.2.3\cdots ..m\right.\right)\right\}. \end{array}$$

A panel of three experts specialized in data mining with bioinformatics have been asked in this stage, with more than five years of experience in this field.

*Data-processing unit*: the opinion matrix refers to the transformation unit's output. The last block begins by using TFNs to turn the opinion matrix into a fuzzy opinion decision matrix. A direct aggregation operator is then applied (i.e., arithmetic mean).  Table 7 illustrates the transform linguistic terms into TFNs after comparing an ideal solution with other values of DM.

^∗^This step used the same Step 4 in the FWZIC methodology.

The best-ranking order correlates to the lowest mean score value.

*External aggregation*: in external aggregation, fuzzy opinion matrices from various DMs are individually processed based on the processes outlined in the processing unit. The outcomes of the decision matrices are then aggregated into the final group decision using the arithmetic mean. In this instance, the expert opinions will be jointed after the final ranking has been determined.

## 3. Result and Discussion

The sequence results for each phase can be presented in this section.

### 3.1. Preprocessing Results

The results of the dataset after imputing the missing value are visualized in Figure 9. The result of SMOTE method is presented in Figure 10. In this context, SMOTE method aid ML models without bias for the diagnosis of ASD.

As shown in Figure 10, the dataset has three balance labels of class “severity”: light, medium, and intense, and each class included 259 instances.

### 3.2. Feature Selection and FWIZC Results

As mentioned in Phase 2, three FS techniques have been applied to the balanced ASD dataset. In addition, the FWIZC method constructed the weights for the medical tests and sociodemographic features within each FS technique.  Table 8 illustrates the results of each technique with its corresponding FWIZC weights.

Table 8 shows that the weights for each set of FS techniques have been obtained based on four physicians' subjective judgments. In this context, the role of the physicians' experience towards feature contributions has been addressed. For the ASD dataset, the relevancies of medical tests and sociodemographic characteristic features have been considered for the severity classes: light, medium, and intense. The benefit of the weighing process is assigning weight to each feature according to its importance. Thus, the constructed hybrid diagnosis ML models in the next section will be designed based on the weighted dataset resulting in a more accurate sense to be closer to reality.

### 3.3. Evaluation Criteria and DM Results

The performance metric results of the 15 hybrid diagnosis models using the developed DM can be shown in Table 9. The 15 models are evaluated using 66% of the dataset for training and 34% for testing.

Table 9 (DM) shows that the 15 models (alternatives) have been evaluated using three performance evaluation metrics (criteria). The hybrid model A1=ReF-decision tree and A6=IG-decision tree have the highest accuracy of 98.94%, while the hybrid model A14=Chi^2^-KNN has the lowest accuracy of 74.30%. Furthermore, many models have similar accuracy results, such as A2=ReF-SVM, A7=IG-SVM, and A12=Chi2-SVM. On the contrary, some models have produced the shortest testing time, zero seconds, such as A1=ReF-decision tree. While A12=Chi^2^-SVM obtained the highest testing time, 1.06 seconds. In addition, A3=ReF-naive Bayes obtained 0.134 seconds for the shortest training time, and A12=Chi^2^-SVM obtained 3.191 seconds for the highest training time. Most ML models have obtained good results concerning the seven performance metrics. All the hybrid models have been measured using weighted datasets resulting from the FWZIC method. Thus, the FWZIC method has provided a suitable guideline for applying the weights to the ASD dataset, increasing the performance metric values. On the other hand, the evaluation results have conflict and trade-off issues among the criteria, making determining the best hybrid model a hard task. Therefore, the evaluation and benchmarking using FDOSM will solve these issues in the next section.

### 3.4. FDOSM Results

As shown in Table 10, there is an overlap of the obtained results for the 15 hybrid models, which cannot provide the precise decision of the best one. So, utilizing the FDOSM to benchmark 15 hybrid models must be achieved to select the best models based on seven evaluation metric criteria. The ranking results for the 15 hybrid models are shown in Table 10 with the score values and orders. The 15 hybrid diagnosis models are ranked according to the score values in ascending order. As the alternative score is lower, the model obtained a better rank and vice versa.

As shown in Table 10, the ranking results of the hybrid models according to the FDOSM reveal that the order of the best/first three hybrid models was A1=ReF-decision tree, A6=IG-decision tree, and A11=Chi^2^-decision tree. In addition, the last/worst three models were A14=Chi^2^-KNN, A9=IG-KNN, and A4=ReF-KNN. A1 is the first-best hybrid diagnosis model for detecting the severity of ASD and obtained a 0.15714 score value, while A6 is the second-best hybrid diagnosis model, obtaining a 0.17539 score value. The third-best rank is the A11 which has obtained a 0.29444 score value. In these contexts, the decision tree classifier has contributed to A29, A47, and A65 to obtain the best diagnosis model and optimal solution for ASD classification. KNN integrates with FS, which performs the lowest diagnosis model for ASD classification.

## 4. Proposal for Future Work

Increasing the opportunities to evidence the risk of medical and behavioral factors in ASD is a valid scientific complex problem where genetic and environmental factors contribute to the emergence of ASD by affecting early brain development. In contrast, apply the FWZIC method to weigh each feature's results. Besides, the intersection of more FS approaches is based on more techniques and more ML. In addition, the use of the new DM consists of eight criteria for performance evaluation metrics, as to utilize the FDOSM method for evaluating and benchmarking large-scale hybrid models to select the optimal model for the diagnosis of ASD.

## 5. Conclusion

This research direction aims at developing a hybrid model through the intersection between nine ML methods and eight FS techniques based on three approaches of FS for predicting and diagnosing autism based on effective sociodemographic and medical by proposing the highest methodological standards applied with high accuracy. Many ML models have been developed to deal with the diagnosis problem from ASD datasets with only sociodemographic features. However, the academic literature does not consider combining medical tests with sociodemographic features to diagnose ASD based on the severity levels. In addition, developing an effective and appropriate ML model for diagnosing autism is important and more reliable, considering the physicians' experience. Therefore, this study considers the literature challenges and overcomes the available issues by combining the ML algorithms, FS techniques, and MCDM methods. Firstly, the methodology developed 15 hybrid diagnosis models using the intersection of three FS techniques and five ML algorithms based on medical tests and sociodemographic features. The FS techniques are Chi^2^, IG, and ReF and are used with the popular supervised ML algorithms decision tree, naive Bayes, KNN, SVM, and AdaBoost. The 15 ML models have been constructed based on a balanced and weighted dataset with the principle of weighing features considering the physicians' experience through the FWZIC method. Since so many developed hybrid models acquired varied metric results, it is difficult to select the optimal model due to conflict and trade-offs between criteria. Therefore, the methodology developed a new DM to evaluate and benchmark all hybrid models using FDOSM based on seven performance metrics: CA, precision, F1 score, recall, test time, train time, and AUC. DM led to the FDOSM method for ranking to select the best optimal model. ReF-decision tree obtained the best rank among all models. The performance metrics for the ReF-decision tree were 0.4190, 0.0030, 0.9946, 0.9902, 0.9902, 0.9902, 0.9902, and 0.9951 for the C1=train time, C2=test time, C3=AUC, C4=CA, C5=F1 score, C6=precision, and C7=recall, respectively. The results demonstrate that the developed methodology reaches flavour performance and surpasses many existing hybrid diagnosis models for autism. The summarized points for this study are as follows:

- Developing these models with the obtained results provides a clear guideline to other researchers on choosing the best ML model supported by scientific justification. Accordingly, the selection process for the best models cannot be achieved based on a specific metric. The performance evaluation metrics should be considered simultaneously for choosing the optimal model within other bioinformatics fields
- To our knowledge, the best hybrid model depends on the expert physicians based on the included and excluded features. More investigation is needed to address this fact through a discussion study with a panel of experts in future work. In conclusion, for the overall results of the three FS techniques, medical test features were less necessary and less beneficial in diagnosing ASD. Most medical features have been excluded, while sociodemographic features have acquired the most important benefits. So, the performance of medical test features affects the diagnosis process less than sociodemographic features. In these contexts, the proposed hybrid model using an MCDM-based ML approach brings up a new concept of applying features' importance as weights when developing the detection model of autism
- An optimal hybrid model resulting from this study increases confidence and encourages global medical users to meet the performance goals of AI applications. These goals can be achieved through the presented evaluation and benchmarking MCDM methodology
- There is one limitation that has been faced in the study. In the FS approach, the process of the selected features is still unclear about how to define a threshold value that represents the stop point for selecting relevant features and excluding irrelevant/few features. Therefore, more experimental research needs to be investigated using more FS approaches to investigate more threshold values

## Figures and Tables

**Figure 1:** Research methodology of evaluation and benchmarking ASD diagnosis models.

**Figure 2:** Percentage of missing values in the ASD dataset.

**Figure 3:** Data imbalance of the ASD dataset.

**Figure 4:** The filter approach.

**Figure 5:** FWZIC methodology of ASD dataset.

**Figure 6:** Membership of TFNs.

**Figure 7:** The intersection process for the developed hybrid diagnosis models.

**Figure 8:** FDOSM Methodology for ASD.

**Figure 9:** Dataset after missing value.

**Figure 10:** Data balance result.

**Table 1:** Description of the real ASD dataset.

No.	Feature name	Medical tests	Sociodemographic	Range	Data type
1	Sex		✓	Male, female	Categorical data
2	The blood type of the patient			A-, A+, B-, B+, O-, O+, AB-, AB+	Categorical data
3	The blood type of the mother	✓		A-, A+, B-, B+, O-, O+, AB-, AB+	Categorical data
4	The blood type of the father	✓		A-, A+, B-, B+, O-, O+, AB-, AB+	Categorical data
5	Relative relation		✓	No, yes	Categorical data
6	Toxoplasmosis	✓		No, yes	Categorical data
7	Unnatural medicines for mother	✓		No, yes	Categorical data
8	Folic acid for mother	✓		No, yes	Categorical data
9	Complications of childbirth for the mother	✓		No, yes	Categorical data
10	Premature baby	✓		No, yes	Categorical data
11	Jaundice	✓		No, yes	Categorical data
12	Smell the food		✓	No, yes	Categorical data
13	Taste the food		✓	No, yes	Categorical data
14	He is afraid of loud sounds		✓	No, yes	Categorical data
15	Degree	✓		609-85	Numerical data
16	Crying for no reason		✓	No, yes	Categorical data
17	Kisses with a sound		✓	No, yes	Categorical data
18	Escaping home when doors are open		✓	No, yes	Categorical data
19	Notice the sound of the bell		✓	No, yes	Categorical data
20	Diapers		✓	No, yes	Categorical data
21	Bathroom skills		✓	No, yes	Categorical data
22	Responds when parents call by name		✓	No, yes	Categorical data
23	Mind wandering		✓	No, yes	Categorical data
24	Vitamin D3	✓		2.90-102.1	Numerical data
25	Vitamin B12	✓		0.01-2050	Numerical data
26	Vitamin zinc	✓		0.9-292	Numerical data
27	Marital relationship for parents		✓	Not good, yes, separate, dead	Categorical data
28	Blood match	✓		No, yes	Categorical data
29	Maternal diseases during pregnancy	✓		No, yes	Categorical data
30	Complications of childbirth for the child	✓		No, yes	Categorical data
31	Chewing food		✓	No, yes	Categorical data
32	Annoying from clothing tag		✓	No, yes	Categorical data
33	Waves		✓	No, yes	Categorical data
34	Patient moving at home		✓	No, yes	Categorical data
35	Patient moves around itself		✓	No, yes	Categorical data
36	Carry out orders		✓	No, yes	Categorical data
37	Laughing for no reason		✓	No, yes	Categorical data
38	Play with children		✓	No, yes	Categorical data
39	Is there a language now?		✓	No, yes	Categorical data
40	Pointing with the index finger		✓	No, yes	Categorical data
41	Notice his name		✓	No, yes	Categorical data
42	Arrange things in one row		✓	No, yes	Categorical data
43	Nodded		✓	Previously, no, yes	Categorical data
44	The age difference between the parents		✓	1-28	Numerical data
45	Duration of premature baby	✓		0-39	Numerical data
46	He plays with circle things		✓	Previously, no, yes	Categorical data
47	Father age		✓	22-83	Numerical data
48	Mother age		✓	16-79	Numerical data
49	Severity (class)	✓		Light, medium, intense	Categorical data

**Table 2:** Five-point Likert scale and equivalent numerical scale.

Linguistic terms	Numerical scoring scale
Not important	1
Slight important	2
Moderately important	3
Important	4
Very important	5

**Table 3:** EDM.

Criteria/experts	*C*1	*C*2	…	Cn
*E*1	$\text{Imp }\left(\frac{E1}{C1}\right)$	$\text{Imp }\left(\frac{E1}{C2}\right)$	…	$\text{Imp }\left(\frac{E1}{\text{Cn}}\right)$
*E*2	$\text{Imp }\left(\frac{E2}{C1}\right)$	$\text{Imp }\left(\frac{E2}{C2}\right)$	…	$\text{Imp }\left(\frac{E2}{\text{Cn}}\right)$
*E*3	$\text{Imp }\left(\frac{E3}{C1}\right)$	$\text{Imp }\left(\frac{E3}{C2}\right)$	…	$\text{Imp }\left(\frac{E3}{\text{Cn}}\right)$
...	…	…	…	…
Em	$\text{Imp }\left(\frac{\text{En}}{C1}\right)$	$\text{Imp }\left(\frac{\text{En}}{C2}\right)$	…	$\text{Imp }\left(\frac{\text{Em}}{\text{Cn}}\right)$

^∗∗^Imp represents the importance level.

**Table 4:** Numerical terms and their equivalent TFNs.

Numerical scoring scale	TFNs
1	(0.00, 0.10, 0.30)
2	(0.10, 0.30, 0.50)
3	(0.30, 0.50, 0.75)
4	(0.50, 0.75, 0.90)
5	(0.75, 0.90, 1.00)

**Table 5:** Fuzzy EDM ($\tilde{\text{EDM}}$) [63].

*Experts*	*Criteria*			
	$\tilde{C1}$	$\tilde{C2}$	*…*	$\tilde{Cn}$
*E1*	$\frac{\tilde{Imp\left(E1/C1\right)}}{\sum_{j=1}^{n}\tilde{Imp\left(E1/C_{1j}\right)}}$	$\frac{\tilde{Imp\left(E1/C2\right)}}{\sum_{j=1}^{n}\tilde{Imp\left(E1/C_{1j}\right)}}$	*…*	$\frac{\tilde{Imp\left(E1/Cn\right)}}{\sum_{j=1}^{n}\tilde{Imp\left(E1/C_{1j}\right)}}$
*E2*	$\frac{\tilde{Imp\left(E2/C1\right)}}{\sum_{j=1}^{n}\tilde{Imp\left(E2/C_{2j}\right)}}$	$\frac{\tilde{Imp\left(E2/C2\right)}}{\sum_{j=1}^{n}Imp\left(E2/C_{2j}\right)}$	*…*	$\frac{\tilde{Imp\left(E2/Cn\right)}}{\sum_{j=1}^{n}Imp\left(E2/C_{2j}\right)}$
*E3*	$\frac{\tilde{Imp\left(E3/C1\right)}}{\sum_{j=1}^{n}\tilde{Imp\left(E3/C_{3j}\right)}}$	$\frac{\tilde{Imp\left(E3/C2\right)}}{\sum_{j=1}^{n}\tilde{Imp\left(E3/C_{3j}\right)}}$	*…*	$\frac{\tilde{Imp\left(E3/Cn\right)}}{\sum_{j=1}^{n}\tilde{Imp\left(E3/C_{3j}\right)}}$
*E4*	$\frac{\tilde{Imp\left(E4/C1\right)}}{\sum_{j=1}^{n}\tilde{Imp\left(E4/C_{4j}\right)}}$	$\frac{\tilde{Imp\left(E4/C2\right)}}{\sum_{j=1}^{n}\tilde{Imp\left(E4/C_{4j}\right)}}$	*…*	$\frac{\tilde{Imp\left(E4/Cn\right)}}{\sum_{j=1}^{n}\tilde{Imp\left(E4/C_{nj}\right)}}$

**Table 6:** DM.

Alternatives/criteria		Performance evaluation metric criteria						
Hybrid diagnosis models		**C1**	**C2**	**C3**	**C4**	**C5**	**C6**	**C7**
A1	ReF-decision tree	C1-A1	C2-A1	C3-A1	C4-A1	C5-A1	C6-A1	C7-A1
A2	ReF-SVM	C1-A2	C2-A2	C3-A2	C4-A2	C5-A2	C6-A2	C7-A2
A3	ReF-naive Bayes	C1-A3	C2-A3	C3-A3	C4-A3	C5-A3	C6-A3	C7-A3
A4	ReF-KNN	C1-A4	C2-A4	C3-A4	C4-A4	C5-A4	C6-A4	C7-A4
A5	ReF-AdaBoost	C1-A5	C2-A5	C3-A5	C4-A5	C5-A5	C6-A5	C7-A5
A6	IG-decision tree	C1-A6	C2-A6	C3-A6	C4-A6	C5-A6	C6-A6	C7-A6
A7	IG-SVM	C1-A7	C2-A7	C3-A7	C4-A7	C5-A7	C6-A7	C7-A7
A8	IG-naive Bayes	C1-A8	C2-A8	C3-A8	C4-A8	C5-A8	C6-A8	C7-A8
A9	IG-KNN	C1-A9	C2-A9	C3-A9	C4-A9	C5-A9	C6-A9	C7-A9
A10	IG-AdaBoost	C1-A10	C2-A10	C3-A10	C4-A10	C5-A10	C6-A10	C7-A10
A11	Chi^2^-decision tree	C1-A11	C2-A11	C3-A11	C4-A11	C5-A11	C6-A11	C7-A11
A12	Chi^2^-SVM	C1-A12	C2-A12	C3-A12	C4-A12	C5-A12	C6-A12	C7-A12
A13	Chi^2^-naive Bayes	C1-A13	C2-A13	C3-A13	C4-A13	C5-A13	C6-A13	C7-A13
A14	Chi^2^-KNN	C1-A14	C2-A14	C3-A14	C4-A14	C5-A14	C6-A14	C7-A14
A15	Chi^2^-AdaBoost	C1-A15	C2-A15	C3-A15	C4-A15	C5-A15	C6-A15	C7-A15

C: criteria; A: alternative; C1: train time; C2: test time; C3: AUC; C4: classification accuracy; C5: F1 score; C6: precision; C7: recall.

**Table 7:** Linguistic terms and their equivalent TFNs.

Linguistic terms	TFNs
No difference	(0.00, 0.10, 0.30)
Slight difference	(0.10, 0.30, 0.50)
Difference	(0.30, 0.50, 0.75)
Big difference	(0.50, 0.75, 0.90)
Huge difference	(0.75, 0.90, 1.00)

**Table 8:** Feature selection results and relevant FWIZC weights.

No.	Chi2-FWIZC weights		IG-FWIZC weights		ReF-FWIZC weights	
1	The blood type of the father	0.015933	The blood type of the patient	0.018751	The patient's blood type	0.016909
2	Vitamin D3	0.015897	The blood type of the mother	0.016847	mother's blood type	0.015103
3	Vitamin B12	0.01408	The blood type of the father	0.016847	Father's blood type	0.015103
4	Jaundice	0.026866	Relative relation	0.015771	m-age	0.028678
5	Marital relationship for parents	0.017665	Vitamin B12	0.014603	f-age	0.016089
6	Patient moving at home	0.033561	Vitamin zinc	0.014603	The age difference between the parents	0.013883
7	Relative relation	0.015516	The age difference between the parents	0.015771	Jaundice	0.025819
8	The blood type of the mother	0.015933	Premature baby	0.026891	Relative relation	0.013883
9	The blood type of the patient	0.017694	Marital relationship for parents	0.022249	Maternal diseases during pregnancy	0.026403
10	Premature baby	0.02585	Blood match	0.021993	Complications of childbirth for the child	0.03063
11	Duration of premature baby	0.024033	Sex	0.027507	Duration	0.022304
12	Sex	0.026708	Unnatural medicines for mother	0.029702	Sex	0.024509
13	Smell the food	0.019389	Taste the food	0.017561	Unnatural medicines for mother	0.026673
14	Taste the food	0.017166	Chewing food	0.014437	Smells food	0.017956
15	Chewing food	0.013635	Annoying from clothing tag	0.019961	Taste the food	0.015681
16	Annoying from clothing tag	0.019389	Waves	0.030499	Chews food before eating it	0.013272
17	Waves	0.028859	Patient moving at home	0.035524	Annoyance with clothing tag	0.017956
18	Patient moves around itself	0.039434	Patient moves around itself	0.041172	Moves around itself	0.037286
19	He is afraid of loud sounds	0.030589	He is afraid of loud sounds	0.031994	He is afraid of loud sounds	0.029177
20	Carry out orders	0.03512	Carry out orders	0.03685	Carry out orders	0.033518
21	Laughing for no reason	0.036231	Laughing for no reason	0.037755	Laughing for no reason	0.034157
22	Crying for no reason	0.027171	Crying for no reason	0.028323	Crying for no reason	0.025705
23	Mind wandering	0.033023	Mind wandering	0.034608	Mind wandering	0.031512
24	Play with children	0.032062	Play with children	0.033915	Mingles with children	0.030955
25	Kisses with a sound	0.015932	Kisses with a sound	0.016912	He kisses the mother by the sound	0.015596
26	Escaping home when doors are open	0.020294	Escaping home when doors are open	0.023215	If he opens the door of the house, he escapes	0.019783
27	Pointing with the index finger	0.033556	Pointing with the index finger	0.039766	Pointing with the index finger	0.031951
28	Notice the sound of the bell	0.025596	Notice the sound of the bell	0.029171	Notice the sound of the bell	0.02424
29	Notice his name	0.032634	Notice his name	0.033905	Notice his name	0.030632
30	Responds when parents call by name	0.023678	Responds when parents call by name	0.024576	Responds when parents call by name	0.022287
31	Diapers	0.020406	Diapers	0.021429	Bathroom skills	0.029392
32	Bathroom skills	0.030423	Bathroom skills	0.032171	Is there a language now?	0.037463
33	Is there a language now?	0.039972	Is there a language now?	0.041533	Arrange things in one row	0.029863
34	Arrange things in one row	0.031764	He plays with circle things	0.032964	Nodded	0.033562
35	He plays with circle things	0.031703	Nodded	0.036986	Marital relationship	0.019868
36	Nodded	0.035259	Duration of premature baby	0.024929	Blood match	0.019786
37	The age difference between the parents	0.015516	Smell the food	0.019961	Toxoplasmosis	0.020299
38	Unnatural medicines for mother	0.028723	Father age	0.018348	Complications of childbirth for the mother	0.02848
39	Complications of childbirth for the child	0.032738			Premature baby	0.024148
40					Diapers	0.019626
41					He plays with circle things	0.029863

**Table 9:** Result of decision matrix.

Alternatives/criteria		Performance evaluation metric criteria						
Hybrid diagnosis models		C1	C2	C3	C4	C5	C6	C7
A1	ReF-decision tree	0.37700	0.00001	0.99312	0.98943	0.98943	0.98944	0.98943
A2	ReF-SVM	2.22900	0.91700	0.95052	0.83245	0.83251	0.83266	0.83245
A3	ReF-naive Bayes	0.13400	0.05000	0.96142	0.84415	0.84367	0.84344	0.84415
A4	ReF-KNN	0.68700	0.51000	0.90306	0.76038	0.74901	0.75549	0.76038
A5	ReF-AdaBoost	0.57700	0.28700	0.98897	0.98528	0.98528	0.98530	0.98528
A6	IG-decision tree	0.47200	0.00200	0.99312	0.98943	0.98943	0.98944	0.98943
A7	IG-SVM	2.70600	0.91400	0.94778	0.83358	0.83364	0.83401	0.83358
A8	IG-naive Bayes	0.21900	0.04000	0.96313	0.84113	0.84029	0.83988	0.84113
A9	IG-KNN	0.60900	0.60600	0.89653	0.75585	0.74503	0.74750	0.75585
A10	IG-AdaBoost	0.69700	0.37600	0.98642	0.98189	0.98189	0.98193	0.98189
A11	Chi^2^-decision tree	0.46600	0.00200	0.99271	0.98830	0.98830	0.98830	0.98830
A12	Chi^2^-SVM	3.19100	1.06000	0.94979	0.83094	0.83080	0.83066	0.83094
A13	Chi^2^-naive Bayes	0.22900	0.04300	0.96235	0.84075	0.83966	0.83926	0.84075
A14	Chi^2^-KNN	0.90700	0.62900	0.89462	0.74302	0.73201	0.73414	0.74302
A15	Chi^2^-AdaBoost	0.75400	0.59500	0.98670	0.98226	0.98226	0.98230	0.98226

C: criteria; A: alternative; C1: train time; C2: test time; C3: AUC; C4: classification accuracy; C5: F1 score; C6: precision; C7: recall.

**Table 10:** FDOSM results of the benchmarking of the 15 hybrid diagnosis models.

Hybrid diagnosis models		Score value	Ranking order
A1	ReF-decision tree	0.157142829	1
A2	ReF-SVM	0.761111002	10
A3	ReF-naive Bayes	0.576984072	7
A4	ReF-KNN	0.781745832	13
A5	ReF-AdaBoost	0.350793653	4
A6	IG-decision tree	0.175396799	2
A7	IG-SVM	0.761111002	10
A8	IG-naive Bayes	0.6007936	8
A9	IG-KNN	0.797618813	14
A10	IG-AdaBoost	0.371428574	5
A11	Chi^2^-decision tree	0.294444441	3
A12	Chi^2^-SVM	0.776983983	12
A13	Chi^2^-naive Bayes	0.6007936	8
A14	Chi^2^-KNN	0.816666435	15
A15	Chi^2^-AdaBoost	0.400000007	6

## Data Availability

Data is available on request (ahmed.bahri1978@iips.icci.edu.iq).
